RETRACTED

# A Novel Approach to Predict Brain Cancerous Tumor Using Transfer Learning

**DOI:** 10.1155/2022/2702328

**Published:** 2022-06-20

**Authors:** Mohammad Monirujjaman Khan, Atiyea Sharmeen Omee, Tahia Tazin, Faris A. Almalki, Maha Aljohani, Haneen Algethami

**Affiliations:** ^1^Department of Electrical and Computer Engineering, North South University, Bashundhara, Dhaka 1229, Bangladesh; ^2^Department of Computer Engineering, College of Computers and Information Technology, Taif University, P.O. Box 11099, Taif 21944, Saudi Arabia; ^3^Software Engineering Department, College of Computer Science and Engineering, University of Jeddah, Jeddah 21959, Saudi Arabia; ^4^Department of Computer Science, College of Computers and Information Technology, Taif University, Taif 21974, Saudi Arabia

## Abstract

As the most prevalent and deadly malignancy, brain tumors have a dismal survival rate when they are at their most hazardous. Using mostly traditional medical image processing methods, segmenting and classifying brain malignant tumors is a challenging and time-consuming task. Indeed, medical research reveals that categorization performed manually with the help of a person might result in inaccurate prediction and diagnosis. This is mostly due to the fact that malignancies and normal tissues are so dissimilar and comparable. The brain, lung, liver, breast, and prostate are all studied using imaging modalities such as computed tomography (CT), magnetic resonance imaging (MRI), and ultrasound. This research makes significant use of CT and X-ray imaging to identify brain malignant tumors. The purpose of this article is to examine the use of convolutional neural networks (CNNs) in image-based diagnosis of brain cancers. It expedites and improves the treatment's reliability. As a result of the abundance of research on this issue, the provided model focuses on increasing accuracy via the use of a transfer learning method. This experiment was conducted using Python and Google Colab. Deep features were extracted using VGG19 and MobileNetV2, two pretrained deep CNN models. The classification accuracy is used to evaluate this work's performance. This research achieved a 97 percent accuracy rate by MobileNetV2 and a 91 percent accuracy rate by the VGG19 algorithm. This allows us to find malignancies before they have a negative effect on our bodies, like paralysis.

## 1. Introduction

Brain tumors are clumps of rapidly developing brain cells that may significantly impair the central nervous system. Additionally, the tumor cell mass might affect the normal functioning of the brain [1, 2]. Additionally, several forms of tumors cause the brain tissue to grow in size over time, resulting in the death of brain cells. Early identification of brain tumors, on the other hand, may significantly improve patients' treatment choices and survival rates. Despite this, manually categorizing tumors using a large number of CT images obtained during normal clinical examinations is a time- and labor-intensive job [3]. Scientists routinely utilize this form of imaging to detect and monitor the growth of brain tumors. CT scans are crucial in the area of automated medical analysis because they visualize the different brain regions and hence give exact information about them [4]. Brain tumors are detected using a variety of imaging modalities, including X-rays, MRIs, and CT scans. The main motivation for this study is to use computed tomography (CT) scans and X-ray pictures to detect brain malignancies. CT scan images are used because they are noninvasive and give extensive information on the size, shape, and location of blood vessels. CT scans are widely utilized because they provide higher-quality images. Scientists have devised a range of ways of identifying and diagnosing brain cancers using CT imaging. These methods include everything from traditional image processing in medicine to advanced machine learning. Deep learning (DL), a subset of machine learning, can learn on its own from both labeled and unlabeled data. In recent years, deep learning approaches and models have shown promise in resolving a variety of complicated issues that need high precision and rely on hierarchical feature extraction and self-learning from data. Pattern recognition, object detection, voice recognition, and other decision-making tasks have all been solved using deep learning [5]. Deep learning, on the other hand, has a major drawback in that it takes a large amount of data to train.

RETRACTED

Without the help of a computer, health professionals would struggle to figure out these huge measurements, particularly more so while undertaking broad information examinations. Moreover, an exact analysis of a dangerous malignant growth might prevent people from acquiring life-saving treatment. For centuries, deep learning strategies have been regularly used to recognize mind growth and surmise different thoughts from information designs. Deep learning has been demonstrated to be suitable for arranging and displaying mind growth. It is a system for finding obscure examples and consistencies in the scope of datasets. It involves a different set of approaches for clarifying the guidelines, standards, and associations that exist inside information groupings, as well as making theories about these associations that might be used to understand recently uncovered information.

Medical care is one of the areas where there is a lack of information when it comes to developing deep learning models using publicly available clinical data. This is, for the most part, because of stress over the protection and security of individual data. As a result, mobile learning has been broadly utilized to overcome information deficiencies in the clinical business. Deep learning, in which a preprepared deep learning model is utilized to handle another issue, is regularly utilized to make up for an absence of reasonable preparation information. The reason for this review is to build a deep learning model for arranging CT outputs and X-beam pictures of cerebrum cancers utilizing move learning. Preprepared deep CNN models, VGG19 and MobileNetV2, are utilized in the proposed model. It is utilized to order CT and X-beam pictures as all things are considered “destructive tumor” or “noncancerous tumor” in light of what it sees.

Various systems for diagnosing and ordering cerebrum growth have been laid out in the literature. Zeineldin et al. [6] proposed a deep brain network-based strategy for sectioning cerebrum growth naturally from attractive reverberation (MR) FLAIR pictures. Their methodology is based on two essential parts: one for encoding and one for unraveling. In the encoder segment, a CNN is utilized to separate spatial data. The resultant semantic guide is then provided to the decoder part, which develops the likelihood map with the full goal. At long last, lingering brain organizations (ResNet) and thick convolutional networks (DenseNet) were investigated. Priyanssh and Akshat [7] used ResNet-50 to fabricate a prescient model for cerebrum cancer discovery by means of machine learning. Their test results showed a 95% accuracy. Nawab et al. [8] discovered a fivefold cross-approval exactness of 94.82 percent using a square-based move learning approach in a comparable study. Their strategy was approved utilizing a benchmark dataset of T1-weighted contrast-upgraded attractive reverberation imaging (CEMRI). Also, Seetha and Raja [9] proposed a computerized approach for identifying mind growth by deep CNN. In the initial step, the Fuzzy C-Means (FCM) technique was utilized to section the cerebrum picture. In another review, Mircea et al. [10] removed wavelet coefficients from pictures utilizing an element-based procedure. Wavelet changes, the creators say, surpass Fourier changes as far as worldly goals go, taking into consideration the obtaining of both area and recurrence data in pictures. The help vector machine (SVM) procedure is then used to make a classifier, which accomplishes 91% precision. At long last, Sujan et al. [11] thought of a method for observing growth in MRI pictures by utilizing a nearby thresholding strategy in view of Otsu's equation and then, at that point, performing the morphological procedure on the MRI pictures. The authors in [12] achieved 86.96 percent accuracy by using the YOLOv5 model. To predict various diseases, various machine learning and deep learning algorithms have been used [13–15].

RETRACTED

The majority of studies that have utilized MRI cerebrum imaging have shown a precision rate of around 90%. But this study presents a comparative analysis of state-of-the-art transfer learning methods for brain cancerous tumor detection. However, the primary goal of this research is to direct exchange picking up using preprepared models and cerebrum CT and X-beam data. Moreover, our research is novel in that we changed MobileNetV2 to get the most significant level of precision (97%), though VGG19 accomplished 91%. In addition, the significant contribution of this study is that it uses and compares two famous transfer learning approaches. This article proposes a strategy for distinguishing cerebral harmful growth by utilizing deep learning. CNN (convolutional neural networking) is a decent methodology for tackling issues of this sort. Using a scope of imaging modalities, this strategy will help in the quick determination of cerebral harmful growth.

As recently expressed, this exploration's key commitment is the execution of three extraordinary exchange learning calculations on a freely open dataset. The segment on results and investigation tends to the execution's results as a whole. The remainder of this exploration is organized as follows. Area 2 examines the technique and materials. Area 3 examines the discoveries and examinations. Area 4 examines the end.

## 2. Method and Materials

The information was taken from the Kaggle dataset, which is openly available to the general population. The assortment included X-beam and CT pictures of both solid and threatening mind growth patients. A CNN is used to separate highlights. The model's four convolutional layers are made up of three Max Pooling 2D levels, one level layer, two thick layers, and a Relu enactment layer. SoftMax, the last thick layer, fills in as an enactment. For the most part, move learning is utilized in this examination to contrast the expected model's precision with the preprepared model's exactness. With minor acclimations to the last layers, preprepared models from MobileNetV2, VGG19, and Inception V3 were utilized, and an ahead model was produced from the essential model. The last layers that are movable include normal pooling, leveling, thickening, and dropout. For separating visual characteristics, the CNN model is viable. The model gathers data from the information contained in photographs and then figures out how to separate them.

RETRACTED

### 2.1. Dataset

This research investigated data on brain tumors that were made publicly accessible [16]. This collection contains photos of brain X-rays and CT scans obtained from individuals diagnosed with a malignant brain tumor. This collection comprises 2513 pictures of individuals with brain cancer and 2087 shots of healthy individuals.

### 2.2. Tools

Python is a strong language for controlling information. Python's expansive library makes deep learning positions easier to execute. A Jupyter Notebook and a Guide were utilized to set up the information. Google Colab was utilized to manage huge datasets and to prepare models on the web as well.

### 2.3. Block Diagram of the System

Figure 1 demonstrates a block design using an X-ray/CT scan image as an input from a dataset split into 2 sections: brain cancer patients and healthy people.

Prior to the preparation of the model, our framework performed numerous preprocessing systems, including procuring pictures of a given size, dividing the dataset, and utilizing information increase strategies. Fitting and tweaking the model brought about better outcomes. To show how misfortune and precision change with age, the disarray grid, model misfortune, and demonstration of exactness have all been shown. Finally, in the event that a client transfers an image as an information model, the result segment might decide if the picture depicts a patient with mental cancer. The square graph is the easiest representation of the total framework. Settling on decisions is a basic part of this framework and is generally explored. Since the model is based on an enormous amount of information accumulated from X-ray pictures, it provides essential assurance.

### 2.4. Preprocessing

Before preparing and surveying the information, preprocessing is performed. The image aspects are resized, the picture pictures are changed over to exhibits, the info is preprocessed utilizing MobileNetV2, and the last advance in every one of the four preprocessing steps is the encoding of hot marks. Scaling a picture is a significant preprocessing step in PC vision since it influences the presentation of the preparation model. It performs all the better when the picture is more modest. The image was extended to 256 × 256 pixels for this examination. The following stage is to change the photos in the assortment into a cluster. The image is changed over to a cluster prior to being utilized on the up and up work. MobileNetV2 involves the image as a pretechnical input. The last advance is to do hot coding on marks since many AI calculations cannot work straightforwardly on named information. This calculation's feedback and result factors should be numeric. For understanding and examination, the labeled information is converted into a mathematical mark.

RETRACTED

In the wake of preprocessing, the information is parceled into three areas: 70% preparation information, 20% approval information, and excess testing information. Individuals who are solid as well as those who have been determined to have a brain disease are displayed in each heap of photographs.

### 2.5. Background of the Proposed Architecture

Convolutional neural networks show the idea of stowed away layers by means of the utilization of brain organizations. Whenever a solitary vector gets an info picture, the brain organization's secret layers direct the scope of brain changes. Each secret layer contains a vast number of neurons, with the preceding layer of each neuron being connected to the following layer of neurons. In contrast, neurons in the same layer are not linked. Every neuron has a unique capability as well as a weighted informational component. Each neuron's output is skewed toward a positive or negative value as a result of the use of capacities and loads. This technique jumps into various secret levels to come up with an end result. The last layer is a completely connected layer that consolidates every one of the covered layers to obtain the eventual outcome. Versatility is a huge weakness of the normal brain organization.  Figure 2 illustrates the proposed design.

Convolutional learning lays the foundation for deep exchange learning. This gathering is entrusted with the obligation of deciding the plan qualities. This layer applies a channel to the source picture. The capacity map is developed through convolution from the results of similar channels. Convolution takes weight ranges and duplicates them according to the information esteem. A channel is made by duplicating a variety of information with a two-layered assortment of loads. When applied to the source and channel, the size of the channel, a dab item delivers a solitary worth. This part goes about as a cradle between the channel and the channel measured patches remembered for the info. The channel is situated beneath the source and is utilized to duplicate a few information sources simultaneously. Since the channel covers the full edge in a calculated style, it is a unique method for recognizing specific kinds of attributes.

The pooling layer sums up the presence of attributes by considering highlight-down inspecting. It is commonly utilized with a convolution layer to accomplish spatial invariance. Separately, normal and maximal pooling are two widely utilized pooling approaches for ascertaining the normal and greatest dynamic presence of a capacity [17]. Without a doubt, the pooling layer takes out unnecessary highlights from the photographs and works on their coherence. The value of the current view is midpointed each time the layer uses normal pooling. When a layer uses normal pooling, it takes the value of its view and averages it. The layer selects the best value in the current channel viewpoint when Max Pooling is enabled. The maximum pooling strategy uses the element guide's picked grid size to pick the very most noteworthy value, bringing about fewer result neurons. As an outcome, the image contracts significantly in size, yet the situation stays unaltered. Pooling is pivotal for reducing the number of component guides and organization boundaries being used. A dropout layer is utilized to forestall overfitting.

RETRACTED

The straightening layer changes the network information over to a one-layered cluster viable with the completely connected layer to make a solitary, one-layered include that is both long and limited in aspect. Vectors might be straightened. At long last, it lays out an association between the single vector and the last order process, alluded to as the “totally associated layer” [18]. All pixel information is remembered as a solitary document, laying out a connection between completely associated layers. The last phases of CNN incorporate straightening and totally connecting layers. It is then changed to a one-layered cluster in anticipation of the resulting completely connected layer of picture classification. CNNs utilize completely associated layers, which have been demonstrated to be extremely worthwhile for picture recognizable proof and grouping in PC vision. The CNN technique begins with convolution and pooling, which disengages and evaluates the picture's key features [18]. Each piece of information is related to a solitary neuron in the layer, and the data sources are straightened. The Relu initiation work is regularly utilized as a totally associated layer. The SoftMax actuation work is utilized to expectably yield pictures in the last layer of the completely associated layer. A completely connected layer is utilized towards the completion of the CNN engineering. This finishes the convolutional brain organization's last couple of layers and most basic layers.

### 2.6. Transfer Learning with MobileNetV2

Clinical scientists face a few obstructions because of an absence of clinical information or datasets. Deep learning strategies are very information-subordinate. Information examination and characterization is a tedious and costly interaction. The advantage of machine learning is that it does not need to bother with an enormous dataset. Estimations become less difficult and more expensive as time passes. Move learning is a technique that involves moving the data acquired from a prepared model on an enormous dataset to another model that needs substantially less information to be prepared. This method began with CNN preparing a little dataset for a particular reason, which incorporated a huge scope dataset that had been recently prepared to utilize preprepared models [19]. Three preprepared CNN-based models were utilized to sort mind X-beam pictures in this review. MobileNetV2, VGG19, and Inception V3 models were utilized. Two kinds of mind X-beam pictures exist: the left one is ordinary, yet the right one has grown. Moreover, this examination utilized an exchange learning approach that is equipped to perform admirably with meager information and is likewise time-effective by utilizing ImageNet information. The system architecture of the transfer learning approach is represented in Figure 3.

RETRACTED

Figure 3 is broken into four significant areas. The primary area gives X-beam photos of the cerebrum. The subsequent part demonstrates how to stack a preprepared model. Three preprepared models are remembered for the subsequent stage. The last stage, as demonstrated in Figure 3, adds the accompanying layers to the stacked, preprepared models. Finally, the result segment isolates the discoveries into two classifications: harmful growth and solid growth.

#### 2.6.1. MobileNetV2

MobileNetV2, a portable convolutional engineering enhanced for mobile phones [20], is a portable convolutional engineering enhanced for cell phones. It depends on altered leftover engineering that uses remaining associations with interface bottleneck levels. Nonlinearity is brought into the transitional expansion layer channels by lightweight profundity and shrewd convolutions. In the MobileNetV2 engineering, a first totally convolutional layer with 32 channels is used, followed by 19 remaining bottleneck layers.  Figure 4 depicts the MobileNetV2 block diagram.

Six phases are expected to create the model: the enhancement picture generator is made; the fundamental model is developed utilizing MobileNetV2, and model boundaries are added; the model is built; the model is prepared, and the model has put something aside for future forecast processes. A deficiency of 0.25 implies that 25% of the loads were taken out arbitrarily throughout the exercise. This strategy brought about a critical decline in the frequency of overfitting. This strategy's significant objective was to keep the model from storing up an exorbitant number of loads and acquiring a broad understanding of the information. This dataset was made with a group size of 32 pictures. As a result, 32 pictures were captured over the span of a solitary cycle. By and large, the model expanded as the clump size rose. In any case, this upsets the model's capacity to sort a few surprising classes. As an outcome, there is a compromise between consensus and particularity when deciding this number. MobileNetV2 is primarily concerned with the presentation of adaptable models in a wide range of model sizes and task types. MobileNetV2 lines are composed of an unending number of rehashing layers [21]. The ordinary state is calculated into profundity shrewd convolution in the portable net through profundity insightful detachable. This needs 11 profundities, an interaction known as pointwise convolution [22].

RETRACTED

### 2.7. Evaluation Metrics

All models were evaluated on the test dataset after the training phase. The performance of these systems was assessed using their accuracy, precision, recall, *F*1 score, and AUC range. The performance indicators for the study are listed below. The number of correctly recognized brain cancer images is represented by true positives (TP), whereas the number of correctly identified normal images is represented by true negatives (TN). The number of correctly recognized normal images as brain cancer images is represented by false positives (FP), and the number of correctly identified normal brain cancer images is represented by false negatives (FN). The confusion matrix is depicted as a block diagram in Figure 5.

The following equations can be derived from the confusion matrix value.

(1) $$\begin{array}{c} \text{Accuracy}=\frac{\text{TP}+\text{FN}}{\text{TP}+\text{TF}+\text{FP}+\text{FN}},\\ \text{ Precision}=\frac{\text{TP}}{\text{TP}+\text{FP}},\\ \text{ Recall}=\frac{\text{TP}}{\text{TP}+\text{FN}},\\ F1=\frac{2\left(\text{Precision}\times \text{Recall}\right)}{\text{Precision}+\text{Recall}}. \end{array}$$

## 3. Result Analysis

For images of normal and malignant brain tumors, we assessed the usability and efficacy of a variety of models and classification methodologies. To classify brain X-ray and CT scan pictures, two pretrained CNN models were used. Both the MobileNetV2 and VGG19 models are viable options. There are two types of brain X-ray and CT scan images. One has a deadly brain tumor, while the other appears to be in perfect condition. The accuracy and loss of a variety of attempted models are summarized in Table 1.

Furthermore, this study employed ImageNet data to implement a transfer learning strategy that works well when only a small amount of data is available for training. Several network topologies, including VGG-19 and MobileNetV2, are explored during the selection process. MobileNetV2 outperformed all other networks, and the findings are based on that architecture.

RETRACTED

### 3.1. Model Accuracy

Figures 6–8 show the findings graphically. In the model depicted in Figure 6, there is no overfitting.

This model is not overfitting because the training accuracy is higher than the validation accuracy, and the validation loss is higher than the training loss.

Train accuracy has increased dramatically after each epoch, as shown by the plot of train accuracy history. The accuracy of the first epoch was 86%, but it improved with each succeeding epoch. The validation accuracy of the model, on the other hand, was 91% and kept growing until the last epoch. A growing line for train correctness has been formed on the model accuracy plot, while a line for test accuracy has been drawn that is continuously between 92 and 97 percent correct over time. Training accuracy is higher than validation accuracy in this scenario (Figure 7).

Here, on the first epoch, the training loss was about 40%, but it gradually decreased until on the final epoch it was less than 10%. Initially, validation loss was also high, but the loss decreased with every epoch (Figure 8).

The accuracy under the curve, or AUC, for training in this case is close to 100%. It is roughly 99.5 percent for validation reasons. Actual values are in columns, while anticipated values are in rows, in the system's confusion matrix. In a classification model, the confusion matrix is used to explain the expected outcomes. The correct and incorrect predictions from the confusion matrix are summarized and categorized. The confusion matrix is depicted in Figure 9.

Here, true positive = 348, true negative = 58, false positive = 2, and false negative = 13.

In this case, MobileNetV2 correctly predicted 406 images and incorrectly predicted 15 images. During testing time, 348 images were classified as healthy and 58 images as cancerous tumors, which is correct. But it predicted 2 images as cancerous tumors and 13 images as healthy, which is not correct.

### 3.2. Model Test

Real-world assessments were also included in this study, which provided data to the system in the form of brain X-ray scans. After the model is built, a file with the extension hdf5 is created that contains the model. For this experiment, three hdf5 files representing three different models were prepared. As a result, a new notebook file with the suffix “ipynb test” is created. Individual X-ray and CT scan images of the brain were used to create this test file, which comprises two models. Figures 10 and 11 show the real-time projections.

Figure 10 shows the output of a malignant tumor in the brain. The model properly predicted an image of a brain malignant tumor based on the input image.  Figure 11 illustrates the input of a typical brain X-ray or CT scan image. Following that, the model returned a good result, indicating that the image submitted by the user depicted a healthy brain.

RETRACTED

### 3.3. Comparison of Result

Table 2 compares our categorization findings to those of the previously stated reference articles.

When compared to previous research that employed comparable pretrained models, VGG19 and MobileNetV2 produced findings that were smooth and accurate from the start. A new study shows that the per-epoch smooth accuracy of VGG19 and MobileNetV2 is much better than that in previous studies. But using the deep learning techniques described [23, 24], they achieved lower accuracy than our proposed model.

## 4. Conclusion

A deep learning scientific structure might be a help for individuals who do not get successive tests or exams in countries with frail medical service frameworks. Deep learning is especially apparent in clinical imaging during early assessments that might suggest deterrent medicine. Because of doctor shortages in resource-limited areas, innovation-aided cerebrum harmful growth recognition is critical for assisting in decreasing the time and exertion spent on cancer distinguishing proof learning-based clinical examination is not quite as astounding as experts would like. This examination recommends that we might have the option to accomplish that degree of exactness by combining different ongoing advancements in deep learning and applying them to pertinent settings. Beginning to end, this exploration utilizes deep figuring out of how to analyze cerebrum cancers. Movable is used to figure out how to prepare a deep CNN with loads preprepared on ImageNet utilizing weighted misfortune work. The brain tumor dataset quantitatively shows the viability of this strategy, with an *F*1 score of 97% and a characterization precision of 99.33 percent on the test set. In the future, the following review will utilize a larger dataset and a greater number of preprepared models. On our dataset, these models performed superbly. MobileNetV2 dealt with these datasets brilliantly. Model approval checked the dependability of the grouping and element extraction results. By utilizing an essential cerebrum picture, these models are fit for distinguishing mind-damaging cancers in the shortest timeframe. X-beam and CT filter innovations are presently broadly available and sensibly valued. As a result, it could be a widely applicable tool for spotting deadly malignancies quickly.

## Figures and Tables

**Figure 1:** Proposed method diagram.

RETRACTED

**Figure 2:** Proposed CNN architecture.

**Figure 3:** Transfer learning system block diagram.

**Figure 4:** MobileNetV2's block diagram.

**Figure 5:** Confusion matrix is depicted as a block diagram.

**Figure 6:** MobileNetV2 training and validation accuracy.

**Figure 7:** Training and validation loss of MobileNetV2.

**Figure 8:** Training and validation AUC of MobileNetV2.

**Figure 9:** MobileNetV2's confusion matrix.

**Figure 10:** Prediction—brain cancerous tumor.

**Figure 11:** Healthy prediction.

**Table 1:** Comparison of different pretrained models.

No.	Configuration	Weighted *F*1 score (%)	Accuracy (%)
1	VGG-19	91.0	91.0
2	MobileNetV2	97.0%	97.33%

**Table 2:** Comparison of accuracy.

This paper model	Model accuracy (%)	Reference paper	Reference paper model accuracy (%)
MobileNetV2	**97.0**	Ref. [23]	85.0
VGG-19	91.0	Ref. [24]	90.28

## Data Availability

The data utilized to support these research findings are accessible online at https://www.kaggle.com/preetviradiya/brian-tumor-dataset.
